# A Robust and Novel Approach for Brain Tumor Classification Using Convolutional Neural Network

**DOI:** 10.1155/2021/2392395

**Published:** 2021-12-21

**Authors:** Tahia Tazin, Sraboni Sarker, Punit Gupta, Fozayel Ibn Ayaz, Sumaia Islam, Mohammad Monirujjaman Khan, Sami Bourouis, Sahar Ahmed Idris, Hammam Alshazly

**Affiliations:** ^1^Department of Electrical and Computer Engineering, North South University, Bashundhara, Dhaka 1229, Bangladesh; ^2^Department of Computer and Communication, Manipal University Jaipur, Jaipur, India; ^3^Department of Information Technology, College of Computers and Information Technology, Taif University, P.O. Box 11099, Taif 21944, Saudi Arabia; ^4^College of Industrial Engineering, King Khalid University, Abha, Saudi Arabia; ^5^Faculty of Computers and Information, South Valley University, Qena 83523, Egypt

## Abstract

Brain tumors are the most common and aggressive illness, with a relatively short life expectancy in their most severe form. Thus, treatment planning is an important step in improving patients' quality of life. In general, image methods such as computed tomography (CT), magnetic resonance imaging (MRI), and ultrasound images are used to assess tumors in the brain, lung, liver, breast, prostate, and so on. X-ray images, in particular, are utilized in this study to diagnose brain tumors. This paper describes the investigation of the convolutional neural network (CNN) to identify brain tumors from X-ray images. It expedites and increases the reliability of the treatment. Because there has been a significant amount of study in this field, the presented model focuses on boosting accuracy while using a transfer learning strategy. Python and Google Colab were utilized to perform this investigation. Deep feature extraction was accomplished with the help of pretrained deep CNN models, VGG19, InceptionV3, and MobileNetV2. The classification accuracy is used to assess the performance of this paper. MobileNetV2 had the accuracy of 92%, InceptionV3 had the accuracy of 91%, and VGG19 had the accuracy of 88%. MobileNetV2 has offered the highest level of accuracy among these networks. These precisions aid in the early identification of tumors before they produce physical adverse effects such as paralysis and other impairments.

## 1. Introduction

A brain tumor is an unregulated and abnormal growth of brain cells. Because the human skull is a rigid and volume-limited body, any unexpected development may damage human functions depending on the brain region involved; additionally, it may spread to other bodily organs, impairing human functions [1]. Brain cancer accounts for less than 2% of all cancers in humans, according to the World Health Organization's (WHO) annual report on cancer, yet it causes massive morbidity and effects [2]. According to Cancer Research UK [3], brain, other central nervous system (CNS), and intracranial tumors kill approximately 5,250 people in the United Kingdom each year. For this reason, the main motivation of this paper is to develop a deep learning-based robust system that can classify brain tumors in a short time. Brain tumor detection is critical in the area of biomedical applications. Recently, the critical nature of brain tumor detection has grown. The brain tumor classification system was created to assist medical personnel in diagnosing the illness. Several methods are required during the classification process, such as preprocessing, feature extraction, and classification. Preprocessing is a step in image processing that occurs prior to doing feature extraction to identify the location of an area or item. Prior to the extraction step, this procedure involves filtering, standardizing, and recognizing items. Feature extraction is the process of extracting fundamental numeric values from images to differentiate them [4].

Without the assistance of a computer, it would be impossible for health practitioners to parse these massive datasets, much more so when doing extensive data analysis. Additionally, a precise classification of a serious tumor may prevent people from receiving necessary treatment. Throughout the centuries, deep learning methods have been extensively utilized to detect brain tumors and infer other concepts from data patterns. The use of deep learning for the classification and modeling of brain tumors is well-known. It is a method for discovering previously unknown regularities and patterns in a wide range of datasets. It includes a broad variety of techniques for exposing rules, paradigms, and relationships within data groupings, as well as for developing hypotheses about these linkages that may be utilized to interpret newly concealed data.  Figure 1 illustrates the primary applications of deep learning in the medical industry.

The use of artificial intelligence (AI) tools in clinical research is rapidly expanding as a result of its accomplishments in prediction and categorization, particularly in clinical analysis to characterize brain tumors, and it is now widely used in biomedical exploration and constructing robust diagnostic systems for various diseases [5–7]. Deep learning (DL) is a subset of machine learning that is typically involving data representations and hierarchical features. For descriptors extraction, DL algorithms use an arrangement of many layers of nonlinear processing techniques. Each successive layer's output becomes the input for the subsequent layer, which aids in data abstraction as we go deeper into the network [8]. Convolutional neural networks (CNNs) are a kind of deep learning that are often employed in visual image analysis and are intended to need little preparation [9]. It is based on the biological functions of the human brain [10] and is used to organize data in a variety of arrays [11]. In the late twentieth century, Lecun et al. built a deep neural network dubbed “LeNet” for use in document recognition applications [12], which was the first use of a deep CNN in a form that was near to its current form. It received a lot of interest after a deep CNN was used to categorize images from (ImageNet LSVRC-2010) using a model called “AlexNet” [13]. AlexNet outperformed other commonly used network topologies during this time period. Following that, its success sparked a string of further triumphs for CNNs in the deep learning field. The primary benefits of CNNs over conventional machine learning and vanilla neural networks are feature learning and infinite accuracy, which can be accomplished by increasing training samples, resulting in a more precise and robust model [14]. Convolutional filters serve as feature extractors in the CNN architecture, and as we go deeper, we extract more complicated features (spatial and structural information). Convolution of tiny filters with the input patterns yields the most differentiating features, which are subsequently used to train the classification network [11].

Over the years, brain tumor categorization has been accomplished utilizing a variety of machine learning methods. In [15], authors proposed a method that combined SVM and KNNfor glioma classification. For multiclassification, an accuracy of 85% is achieved, whereas for binary classification, an accuracy of 88% is acquired. In [16], another approach was proposed for brain tumor detection using Wavelet Transform (DWT), PCA, and ANN-KNN for images classification. The obtained results are between 97% and 98%. Cheng et al. [17] suggested a technique for improving the classification performance of brain tumors by enlarging the tumor area through image dilatation and then dividing it into subregions. They used three ways to obtain features: intensity histograms, GLCM, and BOW, and then combined ring form segmentation and tumor region augmentation to achieve the greatest accuracy of 91.28%. Ertosun and Rubin [18] proposed utilizing CNN to distinguish both low and high grade Gliomas and their grades. They obtained 71% and 96% accuracy, respectively. Paul et al. [19] trained and developed two distinct classification approaches using axial brain tumor images (a fully connected CNN). The accuracy of the CNN architecture, which had two convolutional layers followed by two fully connected layers, was 91.43%. Afshar et al. [20] designed a capsule network (CapsNet) for categorizing brain cancers that considers both the MRI brain picture and the coarse tumor borders. This research had an accuracy of 90.89%. Using CNN and genetic algorithms, Kabir Anaraki et al. [21] suggested two coupled regulatory models for categorizing brain tumor images (GA-CNN). In the first study case, the accuracy for classifying three grades of glioma was 90.9%, whereas the accuracy for diagnosing glioma, meningioma, and pituitary tumors was 94.2% in the second scenario.

Researchers have claimed around 90% accuracy in the majority of studies utilizing MRI brain imaging. However, the main objective of this research is to utilize certain pretrained models for transfer learning using X-ray pictures of the brain. Also, the novelty of this research is that we modified MobileNetV2, and it achieved the highest accuracy of 92%, VGG19 achieved the accuracy of 88%, and InceptionV3 achieved the accuracy of 91%. In this work, a novel method is developed for detecting brain tumors using deep learning. CNN is well-convenient when dealing the current problem thanks to its fast and precise detection of tumors in CT scans.

As mentioned earlier, the main contribution of this research is that three different transfer learning methods have been implemented on a publicly available dataset. All the implementation results have been discussed in the result and analysis part. The remainder of this study is structured as follows.  Section 2 discusses the method and materials; Section 3 discusses the results and analysis; and Section 4 discusses the conclusions.

## 2. Method and Materials

The data were obtained from the free-source Kaggle database. The dataset included X-ray images of both healthy and brain tumor patients. For feature extraction, a CNN is employed. Within the model, there are four Conv2D layers, three Maxpooling2D levels, one flatten layer, two dense layers, and a ReLu activation function. For the last dense layer, the SoftMax is utilized as an activation function. Transfer learning is mostly investigated here to compare the intended model accuracy to the pretrained one. MobileNetV2, VGG19, and InceptionV3 were used for pretrained models, with minor changes in the last layers, and a head model was created from the basic model. Average Pooling, Flatten, Dense, and Dropout are the customizable final layers. The CNN model is useful for extracting visual features. The model extracts the characteristics of the supplied pictures and learns to distinguish the images based on these attributes.

### 2.1. Dataset

This study made use of a publicly accessible brain tumor dataset [22]. This collection contains pictures of brain X-rays from individuals with brain tumors. There are 2,513 brain tumor pictures and 2,087 healthy images in this collection.  Figure 2 shows sample X-ray images for brain tumor and healthy individuals.

### 2.2. Tools

Python is an appropriate tool for data processing especially when dealing with deep learning algorithms. In this study, several Python-based packages are investigated to implement our algorithms.

### 2.3. Block Diagram of the System

Figure 3 shows a block diagram with input as an X-ray picture of a dataset divided into two sections: patients with brain tumors and healthy individuals.

Before training the model, we started by some preprocessing steps involving collecting images, partitioning the dataset, and investigating augmentation methods. The model was fitted and fine-tuned, and the results were improved. The route showing how loss and accuracy vary with epoch has been shown by plotting the confusion matrix, model loss, and model accuracy. Finally, if a user provides a picture as an input to the model, the output section may determine whether or not the image depicts a patient with a brain tumor. The block diagram depicts the complete system in the easiest feasible manner. Making decisions is a critical component in this system and plays a significant role in the research.

### 2.4. Preprocessing

Prior to the data being trained and evaluated, there is a preprocessing phase. Images are resized and transformed to vectors. Then, they are scaled to be suitable for training process. It runs better with a smaller image. 256 × 256 pixels is the resized image in this research. The next step is to process all of the images in the collection into an array. The image is converted to an array for use in the loop function. MobileNetV2 uses the image as a preprocessed input. The last step is the coding. The tagged data are transformed into a numerical label so that it may be interpreted and analyzed. After that, the dataset is splitted into three parts: 70% for training, 20% of validation purpose, and the rest for testing.

### 2.5. Background of the Proposed Architecture

CNNs introduce the idea of hidden layers by using neural networks. When a single vector gets an input picture, the neural network's hidden layers execute a range of neural transformations. Each hidden layer has a huge number of neurons, and the previous layer of each neuron is linked to the subsequent layer of neurons. However, neurons within the same layer are not connected. Each neuron has a distinct function and an input component that is weighted. After functions and weights are applied, each neuron's output is skewed toward a positive or negative value. This method traverses many hidden layers in order to arrive at a conclusion. The final layer is a fully connected layer that mixes all the hidden layers to generate the final result. Scaling is a significant disadvantage in a typical neural network.  Figure 4 shows the proposed architecture.

Deep transfer learning's base layer is the convolutional layer. This is the group that is responsible for deciding the design characteristics. The original image is filtered by this layer. A convolution process multiplies weight ranges with the input. A filter is created by multiplying an array of input data by a 2D collection of weights. A dot product produces a single value when applied to a filter-sized area of the source and filter. This component acts as a buffer between both the input's filter-sized patches and the filter. It is lower than the source and is applied here to multiply several inputs using the same filter. Because it covers the whole frame systematically, the filter is designed as a one-of-a-kind technique for detecting certain types of features.

The pooling layer is used to summarize the characteristics by permitting featured down sampling. Average pooling and max pooling are two extensively utilized pooling approaches that characterize the average existence of a function and its maximum active existence, respectively [23]. Indeed, the pooling layer eliminates superfluous characteristics from the pictures and renders them readable. The layer averages the value of its current view each time it utilizes average pooling. When max pooling is used, the layer picks the largest value from the current view of the filter each time. The max pooling approach picks only the highest value using the matrix size set in each feature map, leading to fewer output neurons. As a result, the picture gets very tiny but the situation stays the same.

The flatten layer converts data from the matrix to a one-dimensional array that may be used in the fully linked layer. Vectors may be flattened. In the last step, the classifier in [24] is applied. When considering CNN, last two stages are flattening and fully connected layers. It is converted to a 1D array in preparation for the next fully connected layer of image classification. Fully connected layers are demonstrated to be particularly helpful for computer vision applications and are largely used in CNNs. The CNN technique's first stages are convolution and pooling, which divide the image down into its constituent features and analyze them separately [25]. Each input is linked to all the neurons in a fully connected layer. In this study, both SoftMax and ReLu activation functions are applied to predict forecast the output. That concludes the CNN's last few layers and most critical layers.

### 2.6. Transfer Learning with MobileNetV2

Analyzing and categorizing big data are expensive and time-consuming processes. To tackle this issue, it is possible to investigate the well-known transfer learning approach which does not necessitate a large dataset to be applied. Calculations become easier and less costly. Transfer learning is a technique that involves using a model that has been trained on a large dataset to transfer its knowledge to a new model that needs to be trained with much less data than required.

Such technique applies CNN on small data [26]. This study included three CNN-based pretrained models to classify brain X-ray images which are MobileNetV2, VGG19, and InceptionV3. Moreover, a transfer learning method, via ImageNet, is investigated to process small data. The investigated architecture for transfer learning is depicted in Figure 5.

There are primarily three distinct sections in Figure 4. The first section contains X-ray pictures of the brain. The second section involves the loading of a pretrained model. Three pretrained models have been loaded in this second section. The third section modifies the loaded pretrained models as illustrated in Figure 4.

#### 2.6.1. MobileNetV2

MobileNetV2 is a mobile-optimized fully convolutional architecture [27]. It is based on an inverted residual architecture, with bottleneck levels linked by residual connections. The intermediate extension layer filters features with lightweight depth-wise convolutions as a source of nonlinearity. A first fully convolutional layer with 32 filters is used in the MobileNetV2 design, which is followed by 19 residual bottleneck layers.  Figure 6 shows the block diagram of MobileNetV2.

Six steps are followed in the development of the model, which creates the amplification image generator, the basic model using MobileNetV2, adds model parameters, builds the model, trains the model, and stores the model for future prediction processes. A loss of 0.25 ensured a random elimination of 25% of the weights during the training. This technique significantly reduced overfitting. The main goal of this approach was to keep the model from utilizing too many weights and from gaining a wide knowledge of the input. For this dataset, a batch size of 32 images was utilized. As a consequence, 32 images were learnt in a single cycle. In general, the model would grow bigger as the batch size increased. However, this reduces the model's ability to classify certain unusual classes. As a result, there is a trade-off between generality and specificity when calculating this number. Over a wide range of model sizes, MobileNetV2 enhances the performance. Every line of MobileNetV2 is made up of *n* times as many repetitive layers [28]. In MobileNet, depth-wise separable is used to factorize the regular state into depth-wise convolution. This entails 11 depth, commonly known as point-wise convolution [29].

### 2.7. Performance Metrics for Image Classification

In this study, several metrices were used to evaluate the performance such as the accuracy, precision, recall, F1-score, and AUC. These measures are based on the following metrics: true positives (TP) determines the number of brain tumor images well identified as tumor images; true negatives (TN) is used to evaluate the number of normal cases which are identified also as normal; false positives (FP) indicates the number of normal images that were incorrectly identified as tumor images; and false negatives (FN) indicate the number of normal tumor images.  Figure 7 shows the block diagram of the confusion matrix.

From the value of the confusion matrix, the following equations can be derived:

(1) $$\begin{array}{c} \text{accuracy}=\frac{\text{TP}+\text{FN}}{\text{TP}+\text{TF}+\text{FP}+\text{FN}},\\ \text{precision}=\frac{\text{TP}}{\text{TP}+\text{FP}},\\ \text{recall}=\frac{\text{TP}}{\text{TP}+\text{FN}},\\ F1\text{-score}=\frac{2\left(\text{precision}\times \text{recall}\right)}{\text{precision}+\text{recall}}. \end{array}$$

## 3. Results and Analysis

We have evaluated the utility and efficacy of many models and methods for classifying healthy and brain tumor pictures. Three CNN models are investigated to categorize brain X-ray images into normal and abnormal which are MobileNetV2, VGG19, and Inception V3. Several alternative network designs are tested throughout the selection process, including VGG19, InceptionV3, and MobileNetV2. MobileNetV2 outperformed all other networks.  Table 1 summarizes the obtained results in terms of accuracy and loss metrics of different models.

### 3.1. Model Accuracy

Figure 8 shows the classification report of MobileNetV2. The F1-score for the classification of healthy and brain tumors is 93% and 91%, respectively.

Everybody can see from the plot of train accuracy history that train accuracy has risen significantly after each epoch. The accuracy was 75% in the first epoch but improved with each subsequent epoch. In comparison, the model's validation accuracy was 84% and grew until the last epoch. On the plot of model accuracy, it can be seen that an increasing line has been formed for train accuracy, while a line has been produced for test accuracy that is consistently between 90% and 96% accurate throughout the period.

Figures 9–11 show the graphical representation of the results. In Figure 9, it shows that the training accuracy is greater than the validation accuracy. Similarly, Figure 10 shows that validation loss is greater than training loss, which indicates that this model has no overfitting issue.

Figure 11 illustrates that the training accuracy under the curve, or AUC, is almost 99%, while for validation, it is almost 98%. The system's confusion matrix is presented, with actual values in rows and predicted values in columns. The confusion matrix summarizes the prediction results in a classification model. The confusion matrix's correct and incorrect predictions are summarized and categorized.  Figure 12 depicts the confusion matrix.

From Figure 11, it has been clear that this model predicted 426 images correctly, but it also predicted 36 images incorrectly.

For qualitative (categorical) items, Cohen's Kappa coefficient (*k*) is a statistic that measures the inter-rater as well as the intrarater reliability. While straightforward % agreement calculations may be more reliable, this method accounts for the potential of agreement arising by coincidence. Using this model, Cohen's Kappa coefficient is 0.84.

### 3.2. Model Test

This study also involved real-world assessment, which fed the model data in the form of X-ray scans of the brain. The real-time predictions are depicted in Figures 13 and 14.

Figure 13 depicts the output of a brain tumor. The model correctly predicted the input image of a brain tumor. On the other hand, Figure 14 shows a healthy brain.

### 3.3. Comparison of Result

In Table 2, we compare our classification outcomes to those of the reference papers mentioned before. With the exception of VGG19, all of the models in Table 2 performed well. When compared with previous studies, this study shows InceptionV3 and MobileNetV2 smooth accuracy per epoch.

## 4. Conclusion

In countries with poor health-care systems, a deep learning analytical framework can be a helpful alternative tool. Deep learning framework for medicine applications shows excellent results especially in early preventive therapy [28, 30–32]. Given that radiologists are in short supply in resource-constrained places, detecting tumors in brain images via advanced deep learning tools can help to minimize effort and speed up the detection process. In this work, we proposed to investigate several advanced deep learning methods and combined them in a new way to increase the expected performance for brain tumor detection. Indeed, we utilize deep learning from start to finish to identify brain tumors. We utilize transfer learning to train a deep CNN with weights pretrained on ImageNet using a weighted loss function. The effectiveness of this approach is shown by quantitative results on the Brain Tumor dataset, which achieves an F1-score of 92% and classification accuracy of 92% on the test set. In the future, work will be done on a bigger dataset and with more pretrained models. In terms of our dataset, these models performed well. With this dataset, MobileNetV2 functioned well. Model verification confirmed that the findings were accurate after classification and feature extraction. Using a simple brain X-ray image, these models can detect brain tumors in the shortest period of time. X-ray technology is now widely available and reasonably priced. As a consequence, it has the potential to be a highly successful technique for brain tumor detection.

## Figures and Tables

**Figure 1:** Primary applications of deep learning.

**Figure 2:** Brain tumor and healthy image.

**Figure 3:** System block diagram.

**Figure 4:** Proposed architecture.

**Figure 5:** System architecture of transfer learning.

**Figure 6:** Block diagram of MobileNetV2.

**Figure 7:** Block diagram of the confusion matrix.

**Figure 8:** Classification report of MobileNetV2.

**Figure 9:** Training and validation accuracy of MobileNetV2.

**Figure 10:** Training and validation loss of MobileNetV2.

**Figure 11:** Training and validation AUC of MobileNetV2.

**Figure 12:** Confusion matrix of MobileNetV2.

**Figure 13:** Prediction-brain tumor.

**Figure 14:** Prediction-healthy.

**Table 1:** Comparison of different pretrained models.

No.	Configuration	Weighted F1-score (%)	Accuracy (%)
1	VGG19	88.18	88.22
2	InceptionV3	90.98	91.00
3	MobileNetV2	92.00	92.00

**Table 2:** Accuracy comparison.

This paper model	Model accuracy (%)	Reference paper	Reference paper model accuracy (%)
MobileNetV2	92.00	Reference [15]	85.00
VGG19	88.22	Reference [17]	90.28
InceptionV3	91.00	Reference [20]	90.89

## Data Availability

The data utilized to support these research findings are accessible online at https://www.kaggle.com/preetviradiya/brian-tumor-dataset.
